The article "Liu Wei Di Huang Wan and the Delay of Insulin Use in Patients with Type 2 Diabetes in Taiwan: A Nationwide Study" was published in 2021. Journal: Evid Based Complement Alternat Med.

# Liu Wei Di Huang Wan and the Delay of Insulin Use in Patients with Type 2 Diabetes in Taiwan: A Nationwide Study

**DOI:** 10.1155/2021/1298487

**Published:** 2021-08-19

**Authors:** Hsin-Hung Chen, Chien-Tung Wu, Yueh-Ting Tsai, Chun-Wei Ho, Ming-Chia Hsieh, Jung-Nien Lai

**Affiliations:** ^1^Intelligent Diabetes Metabolism and Exercise Center, China Medical University Hospital, Taichung, Taiwan; ^2^School of Medicine, Institute of Medicine and Public Health, Chung Shan Medical University, Taichung, Taiwan; ^3^Institute of Traditional Medicine, National Yang Ming Chiao Tung University, Taipei, Taiwan; ^4^Department of Chinese Medicine, Taipei City Hospital, Taipei, Taiwan; ^5^School of Post-Baccalaureate Chinese Medicine, College of Chinese Medicine, China Medical University, Taichung, Taiwan; ^6^Department of Chinese Medicine, China Medical University Hospital, Taichung, Taiwan; ^7^Graduate Institute of Integrative Medicine, China Medical University, Taichung, Taiwan; ^8^Division of Clinical Nutrition, China Medical University Hospital, Taichung, Taiwan; ^9^School of Chinese Medicine, China Medical University, Taichung, Taiwan

## Abstract

**Introduction:**

Patients with type 2 diabetes are widely prescribed metformin for controlling blood glucose levels to avoid related comorbidities. In Taiwan, traditional Chinese medicine (TCM) is also commonly used, especially Liu Wei Di Huang Wan (LWDHW), which has been reported to delay the occurrence of kidney failure. However, the effect of combinational therapy of TCM and oral antidiabetic drugs is still unclear. This study aims to estimate their efficacy in delaying insulin use.

**Materials and Methods:**

This case-control study was conducted using one million randomized samples from the National Health Insurance Research Database in Taiwan. The effects of TCM and LWDHW were estimated using the Cox proportional hazards model.

**Results:**

In this study, 70,036 diabetic patients were enrolled; of them, 17,451 (24.9%) used insulin, while the rest (52,585, 75.1%) did not. TCM users had a lower risk for insulin use (HR: 0.58, 95% CI: 0.56–0.60). LWDHW users had a lower risk compared with patients who used other TCM (HR: 0.86, 95% CI: 0.82–0.90) and presented a dose-dependent effect.

**Conclusion:**

The use of LWDHW and oral antidiabetic drugs is highly associated with the delay in the use of insulin. Clinical practitioners may take them into consideration when treating patients with type 2 diabetes.

## 1. Introduction

Type 2 diabetes is one of the most important noncommunicable diseases in the world. It also poses a public health financial burden on the government because its related comorbidities are 2 to 4 times higher than cardiovascular risk [1]. Diabetes is a well-known complex disease; and many previous studies suggested that earlier multifactorial interventions for diabetic patients could reduce the risks of acute myocardial infarction, stroke, and death. Such is also called the legacy effect of diabetic control [2, 3]. A recent study on five risk factor variables in diabetic patients, namely, elevated glycated hemoglobin (HbA1c) levels, elevated low-density lipoprotein cholesterol levels, albuminuria, smoking, and elevated blood pressure, found that HbA1c level was the strongest predictor of cardiovascular disease (CVD) [4], highlighting the importance of diabetes control. There are many international guidelines with suggested algorithms for comprehensive management of type 2 diabetes, such as lifestyle modification for weight reduction with stepwise pharmacological approaches [5, 6].

The article "Liu Wei Di Huang Wan and the Delay of Insulin Use in Patients with Type 2 Diabetes in Taiwan: A Nationwide Study" was published in 2021. Journal: Evid Based Complement Alternat Med.

Metformin is one of the most commonly prescribed oral antidiabetic drugs (OADs) for type 2 diabetic patients. The intensification of diabetic therapy after metformin, such as additional OADs or insulin, depends on individual characteristics including life expectancy, comorbidities, age, provider and patient's preferences, and the risk of hypoglycemia. However, the majority of diabetic patients in the world did not meet the HbA1c target recommended by the guidelines. One of the reasons suggested in many studies is the clinical inertia of health providers or patients [7, 8]. Clinical inertia would result in avoidance of intensification of diabetic therapy, especially injection with insulin or lack of practice organization to offer or educate the skill of injection [9]. Early intensification of diabetic treatment with insulin was reported to provide significant benefits in both clinical and economic aspects [10]. On the other hand, because diabetes is a progressive disease with a decline in *β*-cell function [11], insulin use is one of the best or optimal choices for diabetic therapy for pancreatic dysfunction. Generally speaking, delayed insulin initiation despite of elevated HbA1c is common [12] due to many reasons including side effects from weight gain or fear of hypoglycemia [13].

Traditional Chinese medicine (TCM) has been widely prescribed for patients in Asia for centuries. In Taiwan, TCM is a form of complementary and alternative medicine usually combined with Western medicine for patients, and this kind of integrative therapy is available under the current healthcare system [14].

Liu Wei Di Huang Wan (LWDHW) is one of the common TCM prescribed for diabetic treatment in Asia [15] and has been reported to delay the development of kidney failure among the type 2 diabetic population [16]. The six ingredients of LWDHW were *Rehmannia glutinosa* (Gaertn.) DC, root, dried; *Dioscorea oppositifolia* L., root, dried; *Cornus officinalis* Siebold & Zucc., fructus, dried; *Alisma plantago-aquatica* subsp. orientale (Sam.) Sam., tuber, dried; Poria cocos (Fr.) Wolf., sclerotium, dried; and *Paeonia x suffruticosa* Andrews, bark, dried. The herbal formulas in the study were prepared as concentrated powders, which were dried to powder after decoction.

The article "Liu Wei Di Huang Wan and the Delay of Insulin Use in Patients with Type 2 Diabetes in Taiwan: A Nationwide Study" was published in 2021. Journal: Evid Based Complement Alternat Med.

Despite the increasing prescription of TCM for type 2 diabetic patients in Taiwan, the long-term evidence of benefits from the combinational therapy of TCM and Western OADs is limited. This study aims to investigate whether combinational therapy delays insulin use in type 2 diabetic patients.

## 2. Materials and Methods

The case-control study was conducted using the National Health Insurance Research Database (NHIRD) in Taiwan. The database was established by the Ministry of Health and Welfare of the Executive Yuan in 1995 and collected all medical records of the National Health Insurance program. The system covered over 99.9% of 23 million nationals and foreigners in Taiwan, which was considered as one of the best health insurance systems in the world.

There are two major medical systems in Taiwan: modern Western medicine and TCM. Both have been practiced in Taiwan for centuries and both are covered by the health insurance system. All prescriptions are collected in the database, which facilitates the analysis of add-on effects of TCM and the drug-herb interaction between TCM and modern medicine. TCM in the current health insurance system includes acupuncture, moxibustion, traumatology, and herbal medicine, also known as internal medicine in TCM. However, the health insurance system does not reimburse herbal medicines in the form of decoction but only covers those in concentrated powders, tablets, and capsules, which are also called Chinese herbal products (CHPs).

The database used in this study contained one million randomized samples, which represent fairly the whole population in Taiwan. After excluding those aged below 20 years, 669,347 adults remained. Of them, 73,787 were recorded as diabetic patients. To ensure that subjects were new insulin users, 3,751 patients who used insulin before 2001 were excluded. Of the remaining 70,036 patients, 17,451 used insulin after the diagnosis of diabetes, while 52,585 did not use insulin. The flowchart of patient selection is shown in Figure 1.

The diseases and treatments in the database were defined according to the International Classification of Diseases, 9th Revision, Clinical Modification (ICD-9-CM) (see Table 1). The medicines and herbs in the database were coded with the number specified by the Ministry of Health and Welfare. The types of antidiabetic drugs were classified with Anatomical Therapeutic Chemical Classification System (see Table 2).

The article "Liu Wei Di Huang Wan and the Delay of Insulin Use in Patients with Type 2 Diabetes in Taiwan: A Nationwide Study" was published in 2021. Journal: Evid Based Complement Alternat Med.

The study period began at the diagnosis of diabetes and ended at the first use of insulin, on December 31, 2012, for cases with no eventual use of insulin. The analysis was conducted using SAS 9.4 (SAS Institute, Cary, NC) with the hazard ratio and 95% confidence interval generated using the Cox proportional hazards model.

## 3. Results

Table 3 shows the demographic data of the patients studied. As can be seen, the gender ratios of insulin users and insulin nonusers were similar, while insulin users were older than insulin nonusers. The prevalence of comorbidities such as hypertension, coronary artery disease, heart failure, stroke, and chronic kidney disease was higher among insulin users, except that of hyperlipidemia. Similarly, more insulin users used diabetic medicines, like thiazolidinedione, sulfonylurea, and metformin, and less users used statins. However, more insulin nonusers chose to take CHPs including LWDHW.

As shown in Table 4, the risk of insulin use decreased with the use of CHPs. Compared with that of CHPs nonusers, the hazard ratio of patients who used CHPs including LWDHW was 0.52 (95% CI: 0.50–0.54), while that of patients who used CHPs excluding LWDHW was 0.58 (95% CI: 0.56–0.60). Similarly, the risk of insulin use for LWDHW users was lower than that of LWDHW nonusers by 0.86 (95% CI: 0.82–0.90).

As shown in Table 5, the effect of LWDHW increased with cumulative dose and cumulative time. Compared with that of LWDHW CHP nonusers, the risk of LWDHW users was significantly decreased when the cumulative dose exceeded 90 grams or the cumulative time was longer than 21 days. The hazard ratios were 0.85 (95% CI: 0.79–0.91) and 0.75 (95% CI: 0.69–0.80) when the cumulative doses of LWDHW were between 90 and 265 grams and above 265 grams, respectively. Moreover, the hazard ratios were 0.86 (0.80–0.92) and 0.71 (0.65–0.76) when the cumulative times of LWDHW use were between 21 and 60 days and longer than 60 days, respectively.

The effects of CHPs in patients who used statins were very similar. As shown in Table 6, compared with that of LWDHW CHP nonusers, the risk of LWDHW users was significantly reduced when the cumulative dose of LWDHW exceeded 90 grams or the cumulative time was longer than 21 days. The hazard ratios of LWDHW users were 0.88 (95% CI: 0.80–0.97) and 0.73 (95% CI: 0.66–0.81) when the cumulative doses were between 90 and 265 grams and above 265 grams, respectively, and were 0.86 (95% CI: 0.78–0.95) and 0.71 (95% CI: 0.64–0.79) when the cumulative times of LWDHW use were between 21 and 60 days and longer than 60 days, respectively.

The article "Liu Wei Di Huang Wan and the Delay of Insulin Use in Patients with Type 2 Diabetes in Taiwan: A Nationwide Study" was published in 2021. Journal: Evid Based Complement Alternat Med.

As shown in Table 7, unlike LWDHW, compared with that of Fang Ji CHP nonusers, the risk of Fang Ji users was not significantly reduced as regards either the cumulative dose or the cumulative time. With Fang Ji as a control herb, the result indicated that the findings of LWDHW cannot be explained by placebo effect.

## 4. Discussion

Analysis results revealed that LWDHW is related to the delay of insulin use in type 2 diabetic patients with dose-dependent effects. To our knowledge, type 2 diabetes is a progressive disease with pancreatic *β*-cell decline or insulin resistance. The characteristics of the diabetic Asian population included increased visceral obesity, impaired insulin secretion, reduced pancreatic *β*-cell mass, young age of diabetes onset, increased microvascular complications, and ischemic stroke. This study attributed the effects of LWDHW on delayed insulin use to stimulation of insulin secretion and enhanced insulin resistance [17].

### 4.1. Insulin Secretion and LWDHW

A Wistar rat study indicated the ability of LWDHW to stimulate insulin secretion and to improve the hyperglycemia condition [18]. The effect on the release of acetylcholine by LWDHW [19, 20] was similar to that of sulfonylurea in augmenting insulin secretion from *β*-cells. *Cornus officinalis*, the major active component of LWDHW, could promote acetylcholine (ACh) release, thus stimulating muscarinic M3 receptors, which could in turn enhance *β*-cell insulin secretion [21]. Another animal research also demonstrated that *Cornus* plays an essential role in decreasing blood glucose levels in an insulin-sufficient state [22]. In other words, LWDHW played a role not only in stimulating insulin secretion, the same as sulfonylurea, but also in stabilizing *β*-cells in diabetic patients. The anti-inflammatory pathway for enhanced insulin sensitivity and protection of *β*-cells might be the possible reasons for delayed insulin use [23].

### 4.2. Insulin Resistance and LWDHW

LWDHW, first reported in Chinese medical literature of the Song Dynasty (1035–1117 CE), is most commonly prescribed in Taiwan. A previous study suggested the benefit of dyslipidemia in patients with metabolic syndrome, implying an association between insulin resistance and LWDHW [24]. An animal study with fructose-rich chow-fed rats showed that *Dioscorea*, one of the components of LWDHW, could reduce insulin resistance and improve insulin sensitivity [25]. Another animal model with obese Zucker rats also showed that LWDHW could delay insulin resistance and increase insulin sensitivity [26]. A possible explanation of the LWDHW effect was the change of insulin action instead of the alternation of insulin secretion. LWDHW could stimulate insulin secretion; and higher insulin levels could enhance the downregulation of insulin receptors [26, 27]. An obese rat model study showed that LWDHW decreased serum triglycerides, nonesterified fatty acid levels, body fat, serum leptin, and insulin levels, suggesting a positive effect of LWDHW in improving insulin resistance [28].

The article "Liu Wei Di Huang Wan and the Delay of Insulin Use in Patients with Type 2 Diabetes in Taiwan: A Nationwide Study" was published in 2021. Journal: Evid Based Complement Alternat Med.

### 4.3. Other Factors between Insulin Delay and LWDHW

In Taiwan, TCM, as a form of complementary or alternative medical treatment, has been widely prescribed together with Western medicine [29]. Such combinational treatment is also covered by Taiwan's National Health Insurance [30]. Previous analysis revealed LWDHW as one of the most common TCM as prescribed for diabetic patients in Taiwan [14]. The convenience to integrate diabetic care with TCM and OADs is an advantage in Taiwan. It improves the clinical inertia of both patients and physicians in diabetes care. Nonadherence could cause poor glycemic control.

### 4.4. Limitations

The National Health Insurance Research Database did not contain laboratory data such as blood glucose level and HbA1c; therefore, we adjusted the complexity of the use of antidiabetic drugs as a poor control of blood glucose level and HbA1c. However, it still lacks lifestyle data such as nutritional status, alcohol consumption, and smoking.

## 5. Conclusion

The integration of TCM/LWDHW and OADs is highly associated with the delay of insulin use, with a significant dose-dependent effect.

## Figures and Tables

**Figure 1:** Flowchart of subject recruitment from National Health Insurance Research Database of Taiwan, 2000–2012.

**Table 1:** International Classification of Diseases, 9th Revision codes.

Diseases or treatments	Codes
Diabetes	250
Dyslipidemia	272
Hypertension	401
Stroke	430–438
Coronary artery disease	410–414
Heart failure	428
Chronic kidney disease	585

**Table 2:** Types of antidiabetic drug.

Drug type	ACT code	Drug name
Biguanides	A10BA	Metformin HCL
		Buformin HCL

Sulfonylureas	A10BB	Glyburide
		Chlorpropamide
		Tolbutamide
		Glibornuride
		Tolazamide
		Glipizide
		Gliquidone
		Gliclazide
		Glimepiride
		Acetohexamide

Combinations of oral blood glucose-lowering drugs	A10BD	Metformin and glimepiride
		Metformin and repaglinide
		Metformin and sulfonylureas
		Metformin and rosiglitazone
		Metformin and pioglitazone
		Metformin and sitagliptin
		Metformin and vildagliptin
		Metformin and saxagliptin
		Metformin and linagliptin

Alpha-glucosidase inhibitors	A10BF	Acarbose
		Miglitol

Thiazolidinediones	A10BG	Rosiglitazone
		Pioglitazone

Dipeptidyl peptidase 4 (DPP-4) inhibitors	A10BH	Sitagliptin
		Vildagliptin
		Saxagliptin
		Linagliptin

Other blood glucose-lowering drugs, excl. insulins	A10BX	Guar gum
		Repaglinide
		Nateglinide
		Exenatide
		Liraglutide
		Mitiglinide calcium hydrate

The article "Liu Wei Di Huang Wan and the Delay of Insulin Use in Patients with Type 2 Diabetes in Taiwan: A Nationwide Study" was published in 2021. Journal: Evid Based Complement Alternat Med.

**Table 3:** Demographic characteristics of subjects with diabetes from National Health Insurance Research Database of Taiwan, 2000–2012.

Characteristics	Insulin users (%)	Insulin nonusers (%)
Total diabetic patients	17,451	52,585
*Sex*		
Male	8,538 (48.9)	25,559 (48.6)
Female	8,913 (51.1)	27,026 (51.4)

*Age (years)*		
Mean ± SD	55.4 ± 13.8	52.7 ± 13.2
<50	6,093 (34.9)	22,672 (43.1)
50–64	6,284 (36.0)	18,986 (36.1)
≥65	5,074 (29.1)	10,927 (20.8)

*Comorbidity*		
Hypertension	4,372 (25.1)	11,866 (22.6)
Hyperlipidemia	2,634 (15.1)	10,062 (19.1)
Coronary artery disease	2,984 (17.1)	8,242 (15.7)
Heart failure	1,115 (6.4)	2,560 (4.9)
Stroke	3,011 (17.3)	7,573 (14.4)
Chronic kidney disease	914 (5.2)	2,615 (5.0)

*Antidiabetics*		
Biguanides	14,000 (80.2)	41,764 (79.4)
Sulfonylureas	14,572 (83.5)	37,808 (71.9)
Combinations	1,991 (11.4)	9,901 (18.8)
Alpha-glucosidase inhibitors	5,410 (31.0)	12,156 (23.1)
Thiazolidinediones	5,618 (32.2)	11,239 (21.4)
DPP-4 inhibitors	1,619 (9.3)	9,207 (17.5)
Others	4,074 (23.3)	8,285 (15.8)

*Complexity of antidiabetics*		
None	2,069 (11.9)	6,111 (11.6)
1 drug	1,332 (7.6)	8,261 (15.7)
2 drugs	4,905 (28.1)	14,972 (28.5)
3 drugs and above	9,145 (52.4)	23,241 (44.2)

*Herbal product usage (days)*		
Never used	9,414 (53.9)	22,715 (43.2)
CHPs without LWDHW	4,486 (25.7)	16,476 (31.3)
LWDHW	3,551 (20.3)	13,394 (25.5)

**Table 4:** Hazard of insulin use of TCM including LWDHW estimated using cox proportional hazards model with National Health Insurance Research Database in Taiwan, 2000–2012.

Herbal product usage	Case/population	aHR (95% CI)	aHR (95% CI)
Total diabetic patients	17,451/70,036		
Never used	9,414/32,129	Reference	
CHPs without LWDHW	4,486/20,962	0.58 (0.56–0.60)	Reference
LWDHW	3,551/16,945	0.51 (0.49–0.54)	0.86 (0.82–0.90)

^*∗*^Adjusted for sex, age, comorbidity, and number of antidiabetics.

**Table 5:** Hazard of insulin use TCM including stratification dose of LWDHW estimated using cox proportional hazards model with National Health Insurance Research Database in Taiwan, 2000–2012.

Herbal product usage	Case/population	aHR (95% CI)	aHR (95% CI)
Total diabetic patients	17,451/70,036		
*Stratified by dose (g)*			
Never used	9,414/32,129	Reference	
CHPs without LWDHW	4,486/20,962	0.58 (0.56–0.60)	Reference
LWDHW < 36	856/3,952	0.55 (0.51–0.59)	0.92 (0.86–0.99)
36 ≤ LWDHW < 90	980/4,380	0.55 (0.52–0.59)	0.93 (0.87–1.00)
90 ≤ LWDHW < 265	904/4,356	0.51 (0.47–0.54)	0.85 (0.79–0.91)
LWDHW ≥ 265	811/4,257	0.45 (0.42–0.49)	0.74 (0.69–0.80)

*Stratified by time (days)*			
Never used	9,414/32,129	Reference	
CHPs without LWDHW	4,486/20,962	0.58 (0.56–0.60)	Reference
LWDHW < 7	622/2,539	0.60 (0.56–0.65)	1.01 (0.93–1.10)
7 ≤ LWDHW < 21	1,277/5,866	0.54 (0.51–0.58)	0.91 (0.85–0.97)
21 ≤ LWDHW < 60	898/4,340	0.51 (0.48–0.55)	0.86 (0.80–0.92)
LWDHW ≥ 60	754/4,200	0.43 (0.40–0.46)	0.70 (0.65–0.76)

^*∗*^Adjusted for sex, age, comorbidity, and number of antidiabetics.

The article "Liu Wei Di Huang Wan and the Delay of Insulin Use in Patients with Type 2 Diabetes in Taiwan: A Nationwide Study" was published in 2021. Journal: Evid Based Complement Alternat Med.

**Table 6:** Hazard of insulin use in statin users of TCM including LWDHW estimated using cox proportional hazards model with National Health Insurance Research Database in Taiwan, 2000–2012.

Herbal product usage	Case/population	aHR (95% CI)	aHR (95% CI)
Total statin users	6,881/34,924		
*Stratified by dose (g)*			
Never used	2,885/14,189	Reference	
CHPs without LWDHW	2,165/11,266	0.69 (0.65–0.73)	Reference
LWDHW < 36	43/2,209	0.63 (0.57–0.70)	0.91 (0.82–1.01)
36 ≤ LWDHW < 90	508/2,468	0.65 (0.59–0.72)	0.93 (0.85–1.03)
90 ≤ LWDHW < 265	472/2,417	0.61 (0.56–0.68)	0.88 (0.79–0.97)
LWDHW ≥ 265	416/2,375	0.52 (0.47–0.58)	0.74 (0.66–0.82)

*Stratified by time (days)*			
Never used	2,885/14,189	Reference	
CHPs without LWDHW	2,165/11,266	0.69 (0.65–0.73)	Reference
LWDHW < 7	314/1,403	0.69 (0.61–0.77)	0.98 (0.87–1.10)
7 ≤ LWDHW < 21	666/3,307	0.64 (0.59–0.70)	0.92 (0.84–1.00)
21 ≤ LWDHW < 60	447/2,401	0.60 (0.54–0.66)	0.86 (0.77–0.95)
LWDHW ≥ 60	404/2,358	0.51 (0.46–0.57)	0.72 (0.65–0.80)

^*∗*^Adjusted for sex, age, comorbidity, and number of antidiabetics.

**Table 7:** Hazard of insulin use in statin users of TCM including Fang Ji as control estimated using cox proportional hazards model with National Health Insurance Research Database in Taiwan, 2000–2012.

Herbal product usage	Case/population	aHR (95% CI)	aHR (95% CI)
Total statin users	6,881/34,924		
*Stratified by dose (g)*			
Never used	2,885/14,189	Reference	
CHPs without Fanɡ Ji	3,924/20,371	0.65 (0.62–0.68)	Reference
Fanɡ Ji < 6	12/50	0.69 (0.39–1.21)	1.04 (0.59–1.83)
6 ≤ Fanɡ Ji < 10.5	21/120	0.49 (0.32–0.75)	0.74 (0.48–1.13)
10.5 ≤ Fanɡ Ji < 26	19/93	0.63 (0.40–0.99)	0.96 (0.61–1.51)
Fanɡ Ji ≥ 26	20/101	0.60 (0.39–0.93)	0.92 (0.60–1.43)

*Stratified by time (days)*			
Never used	2,885/14,189	Reference	
CHPs without Fanɡ Ji	3,924/20,371	0.65 (0.62–0.68)	Reference
Fanɡ Ji < 6	5/33	0.41 (0.17–0.98)	0.62 (0.26–1.49)
6 ≤ Fanɡ Ji < 9	29/146	0.55 (0.38–0.79)	0.83 (0.58–1.20)
9 ≤ Fanɡ Ji < 21	17/81	0.66 (0.41–1.06)	1.01 (0.63–1.63)
Fanɡ Ji ≥ 21	21/104	0.63 (0.41–0.96)	0.97 (0.63–1.48)

^*∗*^Adjusted for sex, age, comorbidity, and number of antidiabetics.

## Data Availability

The data that support the findings of this study are available from National Health Research Institutes, but restrictions apply to the availability of these data, which were used under license for the current study, and so are not publicly available. Data are however available from the authors upon reasonable request and with the permission of National Health Research Institutes.
